# Selenium Status and Its Antioxidant Role in Metabolic Diseases

**DOI:** 10.1155/2022/7009863

**Published:** 2022-07-06

**Authors:** Jing Huang, Ling Xie, Anni Song, Chun Zhang

**Affiliations:** Department of Nephrology, Union Hospital, Tongji Medical College, Huazhong University of Science and Technology, Wuhan 430022, China

## Abstract

Selenium (Se), in the form of selenoproteins, is an essential micronutrient that plays an important role in human health and disease. To date, there are at least 25 selenoproteins in humans involved in a wide variety of biological functions, including mammalian development, metabolic progress, inflammation response, chemoprotective properties, and most notably, oxidoreductase functions. In recent years, numerous studies have reported that low Se levels are associated with increased risk, poor outcome, and mortality of metabolic disorders, mainly related to the limited antioxidant defense resulting from Se deficiency. Moreover, the correlation between Se deficiency and Keshan disease has received considerable attention. Therefore, Se supplementation as a therapeutic strategy for preventing the occurrence, delaying the progression, and alleviating the outcomes of some diseases has been widely studied. However, supranutritional levels of serum Se may have adverse effects, including Se poisoning. This review evaluates the correlation between Se status and human health, with particular emphasis on the antioxidant benefits of Se in metabolic disorders, shedding light on clinical treatment.

## 1. Introduction

The trace element selenium (Se), originally regarded as a toxin, is now recognized as an essential micronutrient [1]. Researchers have found that the Se-containing amino acid selenocysteine (Sec) is the major form of Se in cells. The Sec-containing protein, selenoprotein, is largely responsible for the biological effects of Se [2]. Although selenoproteins are widely expressed in many species, the distribution of selenoproteins varies greatly among species. It has been established that there are 25 genes coding for selenoproteins in the human genome [3]. Most selenoproteins, including glutathione peroxidases (GPx), thioredoxin reductases (TrxR), and iodothyronine deiodinases (DIO) have well-defined oxidoreductase functions, exerting an important role in preventing oxidative injury as an intracellular antioxidant [4]. In addition, several selenoproteins, such as selenoprotein F (SEP15), selenoprotein S (SELS), selenoprotein M (SELM), selenoprotein T (SELT), selenoprotein N (SELN), and selenoprotein K (SELK), are regarded as endoplasmic reticulum- (ER-) resident selenoproteins and are involved in redox sensing and regulation, the unfolded protein response (UPR), and calcium homeostasis [5]. Selenoprotein P (SEPP1), selenoprotein H (SELH), selenoprotein M (SELM), SELT, SEP15, and selenoprotein W (SELW) possess thioredoxin-like domains, suggesting a potential redox-related functions [2]. Selenoproteins represent diverse molecular pathways and biological functions, most notably oxidoreductase functions [2, 3].

In recent years, many studies have shown that the antioxidant effects of Se and selenoproteins have led to great advances in human health and treatment of disease [1, 6–8]. Moreover, the importance of Se supplementation in the prevention and treatment of some diseases has been highlighted. Recently, numerous studies have illustrated the crucial role of Se in chronic metabolic diseases, including cardiovascular disease (CVD), type 2 diabetes mellitus (T2DM), and nonalcoholic fatty liver disease (NAFLD) [9–12]. Previous studies have highlighted the role of excess reactive oxygen species (ROS) in the complex pathogenesis of metabolic diseases [13]. Se, as an antioxidant, shows great potential for redox regulation and the maintenance of cellular homeostasis and metabolism [14]. Many studies have reported that serum Se status is related to the risk of metabolic diseases, and Se supplementation may be a promising approach in patients with low Se levels. In addition, Se levels have been positively associated with blood glucose levels, insulin resistance (IR), and total cholesterol (TC), triglyceride (TG), high-density lipoprotein (HDL), and low-density lipoprotein (LDL) levels, indicating a significant role of Se in glucose and lipid metabolism [15, 16]. Therefore, the protective action of Se, mainly focused on boosting internal antioxidant defense in metabolic diseases, has attracted much attention. However, the molecular mechanism underlying the action of Se in metabolic diseases has yet to be elucidated.

This review summarizes the current knowledge regarding Se status in human health, including Se hierarchy, Se evaluation, Se deficiency, and Se poisoning. Furthermore, we elaborate on the antioxidant properties of Se in the risk of metabolic diseases and from the perspective of Se supplementation trials in the treatment of metabolic diseases.

## 2. Selenium Status in Human Health

Diet is the main source of Se, and approximately 80% of dietary Se is absorbed, depending on the type of food consumed [17]. The Se content in food varies geographically, both within and between countries, and the amount of Se in the diet largely depends on where crops are grown and cultivated, the soil to which animals are exposed, and the foods consumed [1]. Dietary Se is obtained from a wide variety of food sources, including bread and cereals, meat, fish, eggs, vegetables, nuts, milk, and dairy [1, 7, 8]. Knowing the distribution of Se in each food group can provide a basis for dietary recommendations to maintain a Se balance. At nutritional levels, Se is mainly incorporated into selenoproteins, such as SEPP1 and GPx, to exert its biological functions. Studies have shown that dietary Se is mainly absorbed from the duodenum and cecum through a sodium pump via active transport [18]. SEPP1, which accounts for approximately 60% of serum Se, is the major form of Se circulating in the bloodstream. SEPP1 is synthesized and secreted by the liver and transported to other tissues through systemic circulation, and the plasma SEPP1 is absorbed by apolipoprotein E receptor-2 (apoER2) in the brain, testis, and other tissues and by megalin in the kidney (Figure 1) [1, 19–21].

## 3. Se Hierarchy

Although all tissues can synthesize selenoproteins, the amount of Se supplied and the consequences of Se deficiency differ across tissue types. In general, Se is stored in organs and tissues at varying densities: 30% in the liver, 30% in the muscle, 15% in the kidney, 10% in plasma, and 15% in other organs [18]. However, selenoprotein synthesis is regulated by Se availability in the diet. Under conditions of Se deficiency, not all organs or tissues obtain Se equally. In fact, Se retention and redistribution occur in the brain, thyroid gland, testis, and skeletal muscle (SKM), while the levels of Se in the liver, muscle, skin, and other tissues decrease, resulting in the formation a tissue Se hierarchy (Figure 1) [19, 22–24].

As previously reported, the brain expresses all types of selenoproteins [25, 26]. The results obtained from the study of rats fed on a Se-deficient diet showed that while most organs lose up to 90% of Se, the brain retains >75% of Se [27]. Moreover, the thyroid gland is rich in Se and expresses a variety of selenoproteins [28]. Similarly, it was reported that the level of serum Se was decreased in SEPP1-knockout mice, while the thyroid gland morphology, thyroid GPx activity, thyroid Se concentration, and serum levels of thyroid-stimulating hormone (TSH), triiodothyronine (T3), or thyroxine (T4) were all within the normal range, suggesting that low levels of serum Se or SEPP1 do not necessarily interfere with the regular functioning of the thyroid hormone (TH) axis [24]. As for the testes, some studies have indicated that testicular mRNA abundances of GPx4, selenoprotein V (SELV), and TrxR3 are not affected by levels of dietary Se supplementation and were much higher at 6-21 weeks old than at 2 and 104 weeks of age [29]. The total testicular GPx4 level was found to be unaffected in response to diets containing <0.01–5 mg Se/kg, suggesting that selenoproteins in the testis are resistant to the impact of dietary Se levels in order to maintain male reproductive activity [30]. Similarly, neither late nor early developmental disruption of DIO2 in mouse SKM was found to impair muscle function. It is conceivable that, as in the brain and thyroid gland, residual DIO2 in other SKM cells relies on paracrine function and is supplied with sufficient T3 to develop skeletal myocytes in order to maintain SKM function [31–33]. In summary, when Se was deficient, the brain, thyroid gland, testes, and SKM were resistant to Se deficiency (Figure 1). More importantly, selenoproteins in the thyroid were preferentially supplied and even less dependent on serum Se or SEPP1 levels than those in the brain, thyroid gland, and SKM, which indicates the priority of the Se and selenoenzyme supply in the thyroid gland under Se deficiency. On the other hand, previous studies have shown that selenoprotein expression is differentially regulated by Se availability. For example, some selenoproteins (GPx1, SELW, and SELH) are highly regulated by Se availability and belong to the group of stress-related selenoproteins. Other selenoproteins (GPx4, TrxR1, and TrxR3) are less regulated by dietary Se intake and belong to a subclass of housekeeping selenoproteins, indicative of the greatest changes in selenoprotein levels under Se availability conditions [2]. Further studies are required to validate the specific mechanisms that dictate the hierarchy of selenoprotein expression.

## 4. Se Evaluation

At the individual level, Se status can be assessed from hair, toenails, and urinary analyses or blood analysis (including whole blood, plasma, serum, or erythrocyte/platelet fractions) [1]. In general, the level of plasma or serum Se is one of the most used methods for evaluating Se status and intake [34]. For long-term Se status, the toenail and hair Se levels are often employed as markers. Se urinary excretion is closely correlated with plasma and serum levels and can be used to monitor recent dietary intake of Se [34, 35]. Moreover, bioassays of selenoproteins in different blood fractions may provide more accurate estimates of physiological Se status [36]. For example, the concentration of serum SEPP1 is sensitive to dietary Se content; therefore, the level of serum SEPP1 was considered an index of Se nutritional status [37, 38]. However, a high correlation between serum SEPP1 concentration and total Se content in elderly men, young men, and elderly women has been reported, but not in young women, suggesting sexual dimorphism of SEPP1 as a biomarker of Se status in young subjects [39]. Platelet GPx1 and GPx4 activities are recommended as accurate indicators of Se status [40–42]. Burk et al. conducted a randomized controlled trial (RCT) to evaluate the effect of chemical form of Se (sodium selenite, high-Se yeast, and selenomethionine) on plasma biomarkers (Se level, SEPP1 concentration, and GPx activity) and urinary Se excretion in a high-dose human supplementation trial. This study found that supplementation with selenomethionine (SeMet) and Se yeast increased the plasma Se concentration in a dose-dependent manner, but selenite did not [43]. The increased Se levels were related to the amount of SeMet administered. Neither GPx activity nor SEPP1 concentration responded to Se supplementation. Urinary Se excretion was greater after SeMet than after selenite, with excretion after yeast being intermediate and not significantly different from either of the other two [43]. This indicates that plasma Se levels are useful in monitoring the compliance and safety of Se supplementation as SeMet, but not as selenite. Plasma Se levels seem to reflect the SeMet content of yeast but not the other yeast Se forms. As judged by urinary Se excretion, Se in the form of SeMet is better absorbed than selenite [43]. In conclusion, there is a need to select a more appropriate index to reflect the Se status according to specific situations, such as Se deficiency, Se supplementation, individuals, and environmental factors. Further studies are needed to evaluate the strengths and limitations of all potentially available biomarkers of Se measurement in different population groups, including the effects of intake, baseline Se status, duration of intervention, and the possible confounding effects of genotype.

## 5. Se Intake and Diseases

In contrast to many other micronutrients, the intake of Se varies hugely worldwide, ranging from deficiency (associated with Se-deficiency diseases) to toxic concentrations (associated with Se poisoning) [7, 44]. Dietary Se intake ranges from 7 to 4990 *μ*g per day, with mean values of 40 *μ*g per day in Europe and 93 (in women) to 134 *μ*g (in men) per day in the USA [1, 45, 46]. Data from various Asian, European, and Middle Eastern countries show that dietary Se intake and Se status are suboptimal or even low in these populations [47]. The World Health Organization (WHO) indicated that over 40 countries and regions globally suffer from Se deficiency [48]. The recommended dietary allowance of Se ranges from 55 to 70 *μ*g per day, which is typically based on the Se intake needed to saturate GPx activity [49]. However, there is no consensus on a specific cut-off to define Se deficiency, and what is considered a normal range is usually defined based on Se levels in a healthy population in a specific geographical area [50]. Therefore, the minimum requirement for Se intake is to prevent the occurrence of Se-deficient diseases, such as Keshan disease (KD), an endemic cardiomyopathy. The recommended intake of Se has been calculated from the requirement for optimum plasma GPx activity that must, because of the hierarchy of selenoproteins, also consider the amounts needed for normal levels of other biologically necessary Se compounds [50].

## 6. Se Deficiency and Keshan Disease (KD)

KD is a primary endemic cardiomyopathy that only occurs in severely low-Se areas from the northeast to the southwest of mainland China [51]. In other words, the main cause of KD is Se deficiency. Although KD has been effectively controlled in most endemic areas with Se supplementation therapy, chronic and latent KD still exist in some endemic areas with poor economic conditions [52]. Extensive evidence has shown that Se deficiency is strongly associated with KD from an etiological perspective; thus, Se levels are useful for assessing the effectiveness of KD prevention, control, and elimination [1, 7, 51].

Recently, a large and wide scope study, including a total of 6,382 individuals recruited from 1,688 counties in 29 provinces in mainland China, was conducted to explore the role of serum Se and SEEP1 levels in KD. The results showed that Se deficiency may still exist among residents living in some KD-endemic areas, who are still at risk of KD, suggesting the need for a diet rich in Se for the residents in KD-endemic areas [53]. However, the mean serum SEPP1 levels of the residents living in the KD-endemic counties were not significantly lower than those of the residents living in the KD nonendemic counties, which indicated that SEPP1 may not properly reflect the Se status [53]. However, the serum SEPP1 levels in 2,351 subjects living in rural areas, general cities, and developed cities in 15 KD-endemic provinces and 13 KD nonendemic provinces in China were measured [54]. The mean serum SEPP1 levels of residents in KD-endemic areas were significantly lower than those in nonendemic areas, and serum SEPP1 levels were low among individuals in the KD-endemic provinces of Shandong, Inner Mongolia, and Heilongjiang, which indicated that the spatial distribution of SEPP1 was positively correlated with per capita consumption expenditure and soil Se [54]. A local study provided further evidence of SEPP1 as a biomarker for KD [55]. In addition, a spatial ecological study on hair Se levels in KD in Heilongjiang Province, China, showed that the median hair Se levels of the residents in the KD-endemic areas were significantly lower than those in nonendemic areas. Measuring the Se levels in the hair of residents of KD-endemic areas can be a molecular marker of Se nutritional status and provide visualized evidence for the evaluation of KD elimination from the aspect of Se nutrition [56, 57]. Taken together, these data support the idea that Se deficiency is widely accepted as a fundamental cause of KD, and serum Se levels, serum SEPP1 levels, and hair Se levels can be used as biomarkers for monitoring Se status in residents in KD-endemic areas to some degree.

As Se deficiency contributes to the risk of KD, Se supplementation has been proposed to play an important role in the prevention and elimination of KD. In a retrospective long-term follow-up analysis performed on a group of 302 chronic KD patients, 173 (56.3%) of the KD patients were administered Se supplementation until the endpoint of follow-up. Using multivariate analyses, this study clarified that Se supplementation was associated with a decreased risk of cardiac death [58]. Moreover, a randomized double-blind design of children with KD was conducted to assess the relative bioavailability of selenite versus organic Se yeast in a Se-deficient area in China and showed that both forms of Se supplementation (selenite and organic Se-yeast) were equally effective in increasing GPx activity, and Se-yeast provided a longer-lasting body pool of Se [59]. Furthermore, a systematic review and meta-analysis were conducted to evaluate the effectiveness of Se supplementation in the prevention of KD. The administration of Se supplements among the residents of KD-endemic areas significantly reduced the incidence of KD. The protection rates of Se supplements were >80% in 35 studies, and the overall effect (risk ratio) was 0.14 [60]. Therefore, Se supplementation may be a potential strategy for KD prevention and treatment.

## 7. Se Poisoning

Although Se is an essential micronutrient for humans, high levels of Se are harmful, and acute or chronic toxicity resulting from high Se exposure has attracted much attention. Acute symptoms of Se intoxication include abdominal symptoms, such as vomiting, pain, and nausea, as well as garlic breath and cardiac symptoms [61]. Mortality is a serious consequence of acute selenium poisoning. In general, the normal intake levels of Se are between 11 and 280 *μ*g/day [62], the plasma levels of Se are approximately 100 *μ*g/L, and the urinary levels of Se range from 10 to 85 *μ*g/L in the general population [63–65]. Death from Se poisoning has been characterized by plasma Se levels of 300, or as high as 3,000 *μ*g/L, compared to normal levels of 100 *μ*g/L. Nevertheless, individuals with plasma Se levels up to 3,000 *μ*g/L without mortality have also been documented [61]. Similarly, urinary levels of Se related to mortality ranging from 170 to 30,000 *μ*g/L have been reported, and no deaths have been observed in humans with urinary Se levels as high as 1,000 *μ*g/L compared to normal levels of 20–90 *μ*g/L [61]. In recent years, many Se poisoning events have been reported, including large food poisoning incidents and individual dietary poisoning cases.

In 1983–1984, a misformulated Se supplement containing 27,300 *μ*g Se per tablet was taken by 13 individuals, resulting in selenosis symptoms, including abdominal pain, diarrhea, nausea, peripheral neuropathy, fatigue, irritability, hair, and nail changes [66]. Moreover, a March 2008 voluntary market recalls supplement products responsible for the most serious Se toxicity outbreak that occurred in the US, warning consumers that these products caused serious adverse reactions, including significant hair loss, muscle cramps, diarrhea, joint pain, and fatigue, within 10 days of ingestion [66]. The peak levels of Se in these subjects were up to 18.3 *μ*g/g in toenails and 44.1 *μ*g/g in fingernails. Nail samples accurately reflect exposure during this Se toxicity outbreak, which results in long-term or permanent adverse health effects [66]. As for the individual case, a 75-year-old man ingested 10 g of sodium selenite and gradually developed abdominal pain, diarrhea, hypotension, hypokalemia, poor perfusion, and cardiac arrest and ultimately died six hours after exposure [67]. Similarly, a 24-year-old man exhibited typical signs and symptoms of acute Se poisoning, presenting with nausea and vomiting, followed by pulmonary edema and rapid cardiovascular collapse approximately 3 to 4 h after ingestion of a gun bluing agent (likely containing selenous acid). One hour after the suspected ingestion, his serum Se levels reached up to 30,000 *μ*g/L [68]. Moreover, deaths from different types of Se poisoning, such as Se dioxide, selenic acid, and sodium tetraoxoselenate poisoning, are not uncommon [69–71]. In addition, a 51-year-old man and a 44-year-old woman experimented with the daily ingestion of supplement containing Se powder, magnesium powder, zinc drops, and a teaspoon of laxative salts. A few days later, they experienced severe nausea, diarrhea, headache, weight loss, and worsening general condition, as well as considerable diffuse hair loss and white-brownish discoloration of the nails. The serum Se levels in the woman and man were 347 and 387 *μ*g/L, respectively, suggesting a chronic Se poisoning status [72]. Moreover, a previously healthy woman suddenly presented with nausea, vomiting, headache, and dizziness a few days after the ingestion of paradise nuts, as well as massive hair loss after approximately two weeks and discoloration of the fingernails [73]. Detailed diagnostic procedures did not reveal any pathological results, and therapeutic measures did not show any effect. While the thallium and arsenic levels were within the normal range in plasma, the plasma Se levels reached toxic values approximately 8-9 weeks later [73]. This case suggests that we cannot overlook the possibility of Se poisoning in the clinical diagnosis.

In summary, although acute or chronic Se poisoning is rarely observed, its consequences can be serious and even fatal. Thus, attention must be paid to foods with a high Se content to avoid eating too much by mistake. Studies on the Se content in humans have revealed that toxic effects occur following a daily intake of at least 300 *μ*g [72]. In addition, noncritical Se intake without a physician's recommendation should be urgently dissuaded. As a part of the therapeutic strategy, there is a need to consider its limited therapeutic range to avoid overdose and related toxicity.

## 8. Se Levels and Metabolic Diseases

Prospective studies have found that a high Se status is associated with decreased mortality, wherein low plasma Se was related to increased overall and cancer mortality [74–76]. Moreover, Se levels were also associated with the incidence of new-onset heart failure, anemia, iron deficiency, high C-reactive protein (CRP) levels, and current smoking [74]. Recently, it was reported that serum Se is related to multiple indicators of metabolic syndrome, including high levels of blood glucose, cholesterol, and body mass index (BMI) in the general adult population [74]. For instance, a cross-sectional analysis of 4,339 participants found that Se levels were positively associated with IR and blood glucose; that is, a 10 *μ*g/L increase in Se was associated with a 1.5% increase in insulin [15]. On the other hand, a large cross-sectional study of 8,198 rural Chinese reported that serum Se levels were positively correlated with total cholesterol (TC), TG, HDL, and LDL, and elevated serum Se levels were related to an increased risk of dyslipidemia, which indicated the crucial role of Se status in lipid metabolism [16]. These studies indicate that high levels of Se are associated with IR and dyslipidemia. Therefore, it has been proposed that the relationship between Se status and various health outcomes, especially in metabolic diseases, requires close attention. In summary, these results indicate the relevance of Se status in public health. Understanding the association between Se status and human health is essential for developing effective public health policies, guiding applicable clinical practice, and counteracting health issues associated with Se deficiency.

Due to the antioxidant activity of Se, its protective role in metabolic diseases, including coronary heart disease (CHD), HT, T2DM, and nonalcoholic fatty liver disease (NAFLD), has been previously demonstrated [1, 6, 8, 77]. In addition, considering the crucial role of Se in the cellular antioxidant defense system, therapeutic strategies involving Se supplementation for the treatment of certain diseases have been underway for many years [77, 78]. Recently, this practice has achieved promising results in the prevention and treatment of metabolic diseases, including CHD, HT, NAFLD, and T2DM [6, 79–82].

## 9. Coronary Heart Disease (CHD)

Coronary atherosclerotic heart disease is caused by the narrowing or occlusion of the vascular lumen due to coronary atherosclerosis (AS), which eventually leads to myocardial ischemia, hypoxia, or necrosis, also known as CHD [83]. Oxidative stress, endothelial dysfunction, hyperlipidemia, and inflammation are involved in the pathogenesis of AS. As an antioxidant agent, several prospective investigations have declared the association between Se level and cardiovascular risk and outcomes [1, 2, 7].

Recently, a meta-analysis compared the Se levels between CHD patients and healthy individuals and found that the level of Se was lower in CHD patients than in healthy individuals, indicating that Se status may have some effect on the risk of CVD [84]. A nested case-control study of 1,621 CHD cases in the prospective Dongfeng-Tongji cohort also found that CHD risk was inversely associated with plasma Se levels [85]. Another meta-analysis, including 25 observational studies, further clarified that a 50% increase in Se level was associated with a 24% reduction in CHD risk in observational studies, suggesting an inverse correlation between Se levels and CHD risk [86]. Moreover, a meta-analysis including 16 prospective observational studies showed a nonlinear relationship between CHD risk and blood Se levels across a range of 30-165 *μ*g/L and a significant benefit of CHD within a narrow Se range of 55-145 *μ*g/L [87]. In a small Chinese cohort study of 1,103 cohort participants, the inverse association between CHD mortality and serum Se level was 73 *μ*g/L [88]. In addition, a study using data collected from 17,867 individuals showed a U-shaped association between dietary Se intake and all-cause mortality, wherein the serum Se levels were negatively but nonlinearly associated with the incidence of CHD [89]. These analyses highlight the significant benefit of higher levels of Se in the prevention of CHD. Furthermore, several selenoproteins play vital roles in the heart; for example, low Se levels disrupt the synthesis of a subgroup of stress-induced selenoproteins, including GPx1, leading to a shortage of one or more of these crucial proteins in the heart [90]. A case-control study on 85 CHD patients indicated a reduction in GPx1 activity related to increased CHD severity, which suggested that GPx1 activity may be a useful marker for predicting and monitoring CHD [91]. In summary, Se status and GPx1 are tightly related to the incidence and mortality of CHD. Additional research is needed to confirm whether Se may attenuate the adverse effects of CHD and to investigate the potential underlying mechanisms.

Based on the inverse relationship between Se levels and CHD risk, moderate Se supplementation may be beneficial in preventing CHD risk. Among six RCTs, including a total of 17,766 participants, four trials used Se supplementation combined with other vitamins or minerals, while two trials used Se supplementation alone. Se supplementation was found to result in a nonsignificant 11% reduction in coronary events, as the trials were small and Se was administered in combination with other vitamins or minerals in all but two trials [86]. Another RCT illustrated that probiotic and Se cosupplementation had a favorable effect on glucose and lipid metabolism and anti-inflammatory and antioxidant capacity, compared with placebo in CHD [92]. Moreover, a five-year prospective RCT among 443 Swedish citizens aged 70–88 years showed that the combined supplementation of Se and coenzyme Q10 significantly reduced CVD mortality, accompanied by a decreased level of N-terminal pro-BNP and a better cardiac function score, compared with the placebo group [93]. Even after 12 years, CVD mortality was significantly reduced in the actively supplemented group, as well as in subgroups of patients with diabetes, HT, ischemic heart disease, or impaired functional capacity, compared with the placebo group [94]. These results suggest that the protective action of Se supplementation was not confined to the intervention period but persisted during the follow-up period [94]. Alehagen et al. further indicated that supplementation with Se and coenzyme Q10 resulted in lower concentrations of both copeptin and MR-proADM (as oxidative stress biomarkers) in a four-year prospective RCT among 437 elderly Swedish citizens [95]. A secondary analysis of this RCT showed a decreased level of CRP and sP-selectin (as inflammation biomarkers) in the active supplementation group compared with the placebo group, indicating a significant effect of Se on inflammation and AS [96]. Recently, Alehagen et al. used structural equation modelling to explain the underlying mechanisms of the protective action of Se in CVD and found that Se supplementation reduced inflammation and oxidative stress, which reduced myocardial fibrosis and improved myocardial function [97]. However, a meta-analysis including 16 RCTs with 43,998 participants reported that Se supplementation significantly lowered serum CRP levels and increased GPx activity but had no effect on CHD mortality and lipid profile [98]. Another study showed that oral Se supplements (200 *μ*g/day) for two weeks to 144 months significantly increased blood Se levels by 56.4 *μ*g/L, whereas oral Se supplements (100 *μ*g/day) for 6–114 months had no effect on CHD, suggesting that Se supplementation had no effect on CHD [87]. Although the results of these clinical trials are not entirely consistent and need to be further studied, evidence from animal studies suggests that Se may protect against experimental AS. In the apolipoprotein E-deficient mouse model of AS, dietary SeMet supplementation increased Se levels and GPx activities, reduced lesion burden and inflammatory response, and improved vessel function compared with the nonsupplemented group [99]. Xiao et al. also showed consistent results that oral administration of both Se nanoparticles (SeNPs) and Na_2_SeO_3_ for 10 weeks significantly reduced AS lesions in mouse aortae by alleviating vascular endothelial dysfunction [83]. In summary, few RCTs have addressed the efficacy of Se supplementation on CHD risk, and their findings remain inconclusive. The preliminary results of studies conducted on animal models may not truly reflect the effectiveness of Se supplementation in preventing or treating CHD; evidence from large RCT is needed to confirm the feasibility of Se supplementation as the treatment therapy for CHD.

## 10. Hypertension (HT)

HT is a cardiovascular syndrome that is characterized by elevated systemic arterial pressure. Oxidative stress, inflammation, and endothelial dysfunction are considered the major pathological factors associated with HT [100]. Some studies have shown that individuals with HT can produce more ROS and have an impaired antioxidant defense system, both of which increase oxidative stress and lead to an ongoing vicious cycle [101]. ROS, in turn, activate chemoreflex and suppress baroreflex, thereby stimulating the sympathetic nervous system and causing HT [102]. Se, an essential micronutrient with antioxidant properties, has been hypothesized to play a protective role against HT.

Xie et al. conducted a 20-year cohort study and found that the cumulative intake of Se was inversely associated with the risk of HT only in northern residents (low-Se zone), but not in southern residents, suggesting that the association between Se intake and the risk of HT varied according to regions in China [80]. A 10-year prospective study conducted in South Africa found that baseline Se levels were negatively associated with blood pressure (BP), indicating a vascular protective effect of Se [103]. Furthermore, in low soil Se zones, high Se intake may be beneficial for the prevention of HT, as low Se levels are associated with left ventricular hypertrophy, which is the main pathological change leading to HT [104]. Recently, Wang et al. conducted a secondary analysis and inferred a significant inverse association between plasma Se levels and HT risk [105]. These studies suggested that low Se levels were a risk factor for HT; however, opposing findings have since been reported. For instance, a cross-sectional study of 9,076 urban and rural residents in Shandong Province of China indicated that higher Se levels were associated with an increased risk of HT in women, but not in men, by logistic regression analysis, suggesting that high Se levels in women were more likely to increase the risk of HT compared to similar levels in men [106]. Another cross-sectional study concluded that chronic overexposure to environmental Se elevated BP, particularly in women [107]. Moreover, a longitudinal study on 2,000 elderly individuals indicated that higher Se levels were associated with higher BP and HT risk [108]. Surprisingly, these studies showed that high Se levels may play a harmful role in the prevalence of HT, which is in contrast to the results of previous studies. In contrast, in a cross-sectional study in China, high environmental Se exposure increased the prevalence of HT, but there was no significant association between Se level and the risk of HT [109]. Tan et al. reported a U-shaped association between serum Se levels and all-cause or cardiovascular mortality in patients with HT [110]. The nadir mortality of all-cause and cardiovascular events occurred at serum Se levels of 136 and 130 *μ*g/L, respectively [110]. In conclusion, the correlation between Se levels and HT risk remains unclear. Whether positive, negative, or U-shaped, further studies, especially large RCTs, will be needed to address these contrasting results.

Considering the controversial role of Se in HT, the potential benefit of Se supplementation on the risk of HT remains to be elucidated. Currently, no RCTs have been published wherein Se supplementation is the sole intervention for HT. However, cosupplementation in Se-depleted areas has been shown to reduce the risk of gastric cancer, stroke, and overall mortality, but not in HT and CVD [111]. In addition, a larger RCT that cosupplemented Se with *β*-carotene or *α*-tocopherol also showed no difference in BP compared to control groups [112]. Moreover, various studies have shown that increasing Se levels above the recommended daily intake are not beneficial and lead to HT, diabetes, and hyperlipidemia [113]. In summary, additional experimental evidence and RCT data are needed to gain further insights into the role of Se in the risk of HT, particularly to clarify the underlying mechanisms. The application of Se supplementation for the prevention of HT requires further discussion.

## 11. Nonalcoholic Fatty Liver Disease (NAFLD)

NAFLD, including simple steatosis (NAFL) and nonalcoholic steatohepatitis (NASH), is the most common cause of liver disease worldwide, and its incidence is increasing in parallel with obesity and diabetes [114]. NAFLD is a complex disease that is modulated by numerous mechanisms, including metabolic, genetic, and gut microbial factors [115]. Some injurious processes, such as oxidative stress, UPR response, and lipotoxicity, contribute to liver damage, progressive fibrosis, and cirrhosis [114]. Owing to the role of Se in lipid metabolism and antioxidant defense, extensive evidence has suggested that Se may contribute to the development of NAFLD.

Recently, a cross-sectional analysis of 3,827 adults without viral hepatitis, hemochromatosis, or alcoholic liver disease indicated a nonlinear association between serum Se levels and alanine aminotransferase (ALT) activity and NAFLD risk [81]. These positive associations were only found above a serum Se level of 130 *μ*g/L, whereas no association was observed below this value [81]. Another large cross-sectional study of 8,550 adults in China demonstrated that increased plasma Se levels were associated with an increased risk of NAFLD, which may be mediated by IR and oxidative stress [116]. In addition, this study found that elevated plasma Se levels were related to higher TG, LDL, ALT, aspartate aminotransferase (AST), gamma-glutamyltransferase (*γ*-GT), fasting plasma glucose, postloading plasma glucose, and IR [116]. However, previous studies have shown that Se levels are low in patients with NAFLD and cirrhosis. Reja et al. reported an inverse relationship between serum Se levels and the risk of advanced liver fibrosis, indicating that Se may be beneficial for the prevention of liver fibrosis in the development of NAFLD [117]. In contrast, several animal studies have indicated that Se exposure could induce increased serum liver enzyme levels, the activation of Kupffer cells, and higher hepatic IR and TG levels in animals, suggesting that Se exposure may be associated with the development of NAFLD [116]. Regarding the role of selenoproteins in NAFLD, Day et al. performed a transcriptomic exploration of the expression of selenoproteins in NAFLD and healthy individuals. Bioinformatics analysis revealed lower levels of TrxR3 and SELO expression in NAFLD, while SELM, DIO1, GPx2, and GPx3 were highly expressed in NAFLD compared with the healthy group [118]. A case-control study showed that SEPP1 levels were positively correlated with NAFLD risk factors including BMI, ALT, AST, and *γ*-GT. In addition, the overexpression of SEPP1 aggravated lipid accumulation and inhibited AMPK/ACC phosphorylation, providing insights into SEPP1 in the diagnosis and treatment of NAFLD [119]. Caviglia et al. also clarified a close association between SEPP1 levels and altered metabolic profiles and degree of hepatic fibrosis [120]. However, whether Se levels are positively or negatively associated with NAFLD risk in humans remains unclear. Thus, the importance of selenoproteins in NAFLD cannot be ignored, and further research is needed to demonstrate the precise role of Se in NAFLD.

Although the specific role of Se in NAFLD remains unclear, few studies have investigated the effects of Se supplementation in NAFLD patients. In animal experiments, feeding NAFLD mice with Se for four months decreased AST and ALT activity, hepatic damage-associated diagnostic markers, and serum lipid levels, suggesting a protective role of Se supplementation in NAFLD [121]. Another animal experiment found that Se supplementation had a beneficial effect on hepatic injury in mice [122]. Recently, Wang et al. found that Se supplementation was beneficial for alleviating hepatic injury and IR during NAFLD, which was mediated by activating the KEAP1/NRF2 pathway [123]. In conclusion, animal studies have indicated that Se supplementation may be a potential therapy for the prevention and treatment of NAFLD. However, these preliminary experiments conducted on animal models may not truly reflect the specific value of Se supplementation in clinical trials. Therefore, further clinical trials will be needed to elucidate the role of Se supplementation in patients with NAFLD.

## 12. Type 2 Diabetes (T2DM)

T2DM is characterized by hyperglycemia, IR, and a relative decrease in insulin secretion, which often occurs in younger individuals [82]. The pathogenesis of T2DM is complex, and IR and *β* cell failure are two core pathophysiological defects in T2DM. Redox imbalance can provide a reasonable explanation for the occurrence and progression of T2DM [124]. Recently, several studies have reported that elevated ROS levels in pancreatic *β* cells are associated with elevated fasting plasma insulin levels and the absence of IR, resulting in pancreatic *Β* cell dysfunction and subsequent progression to T2DM [102]. Moreover, intracellular ROS accumulation causes defective angiogenesis in response to ischemia, activates a number of proinflammatory pathways and genes, and inactivates antiatherosclerosis enzymes, resulting in the development of diabetes complications, such as AS and cardiomyopathy, which is caused in part by pathway-selective IR [125]. Thus, increased superoxide production is the central and major mediator of diabetic tissue damage. Based on the role of Se in glucose metabolism and antioxidant defense, Se may be involved in the pathogenesis of T2DM [126].

Several studies have demonstrated the importance of Se in T2DM patients. A case-control study showed that T2DM patients had higher levels of Se than healthy individuals [126]. A case cohort study also found that higher serum Se levels were associated with an increased risk of T2DM [127]. In a meta-analysis, eight observational studies demonstrated a statistically significant positive association between Se levels and the risk of T2DM [82]. Similarly, a linear association between plasma Se level and T2DM risk was observed in a Spanish study [128]. Moreover, a prospective cohort study in Italy showed that higher dietary Se intake increased the risk of the first hospitalization for T2DM [129]. Although many studies have reached a consensus that high Se exposure is a risk factor for T2DM, the relationship between dose and effect remains unclear. Thus, Vinceti et al. conducted a meta-analysis of 34 nonexperimental studies and found a direct relationship between Se exposure and T2DM risk. As a result, a clear and roughly linear trend was observed in subjects with a higher serum Se level of 140 *μ*g/L. At Se levels up to 160 *μ*g/L, the risk ratio was as high as 1.96, indicating a dose-response association between Se exposure and T2DM [130]. In contrast, serum Se levels have been reported to be positively correlated with insulin levels and IR markers [15]. Regarding the role of selenoproteins in T2DM, SEPP1 was highly expressed in T2DM patients, leading to IR by eliminating physiological ROS required for insulin signal transduction [131]. Mita et al. isolated SEPP1-neutralizing antibodies that improved glucose tolerance, IR, and insulin secretion in a T2DM mouse model, suggesting that elevated SEPP1 levels are an effective target for T2DM treatment [132]. A prospective study in the Japanese population even indicated that SEPP1 may be a marker for predicting hyperglycemia [133]. These studies clarified that the association between serum Se and T2DM may depend on the upregulation of hepatic SEPP1 biosynthesis under IR and hyperglycemia conditions [134]. Similarly, SELS is involved in the pathogenesis of T2DM through inflammatory responses, oxidative stress, and ER stress [135]. Taken together, these results highlight the significant role of Se and selenoprotein in T2DM. However, the relationship between Se and T2DM varies in RCTs and observational studies, and its specific role and mechanism have yet to be fully elucidated.

With respect to the contributing factor of Se in T2DM, it is worth exploring whether Se supplementation can increase the risk of T2DM. A meta-analysis showed that Se supplementation increased the risk of T2DM by 11% compared with placebo, with a higher risk ratio in women than in men [130]. In addition, an RCT on 54 patients with T2DM and CHD found that probiotics and Se cosupplementation improved mental health parameters and metabolic profiles in T2DM patients [92]. In contrast, some studies have reached inconsistent conclusions. To examine the effect of long-term Se supplementation on the prevalence of T2DM, a secondary analysis of 1,202 subjects without T2DM at baseline was performed [136]. During an average follow-up of 7.7 years, Se supplementation had no effect on the risk of T2DM in analyses stratified by age, sex, BMI, and smoking status [136]. Similarly, Stranges et al. reported that there was no significant change in HbA1c in an elderly European population with a low Se status after 2 years of Se supplementation [137]. Moreover, a meta-analysis of RCTs indicated that a higher risk of T2DM was not observed in the Se supplementation group compared to the placebo group [82]. A systematic review of RCTs also found no evidence to support the increased risk of Se supplementation in T2DM [138]. These studies suggest that Se supplementation does not increase the risk for T2DM. These inconsistent results may be explained by a possible U-shaped response of Se supplementation to glucose metabolism [137]. Overall, further longitudinal, cross-sectional studies and RCTs are needed to demonstrate whether Se supplementation can increase the prevalence of T2DM to further verify whether high Se levels are a risk factor for T2DM.

## 13. Conclusions

As an important microelement, Se is mainly obtained through the diet, including via supplements, absorbed from the duodenum and cecum, and transported to various tissues in the form of SEPP1 (Figure 1). It mainly exerts its nutritional and antioxidant activities on human health and diseases in the form of selenoproteins. Given the antioxidant defense of these selenoproteins, Se has been used to mitigate oxidative stress in multiple diseases, including CVD, T2DM, thyroid disease, neurodegeneration, infection, infertility, and cancer (Figure 2). Recently, extensive evidence has been reported that supports the significant role of Se in the prevention, onset, and clinical outcomes of metabolic diseases, such as CVD, HT, NAFLD, and T2DM. Herein, we review these studies, focusing mainly on the last 20 years of research. According to the reported data, a close correlation between Se status and favorable prognosis of the abovementioned pathologies has been generally observed. Se supplementation has been widely studied as a therapeutic approach for the prevention of metabolic diseases, delaying the progression, and alleviating the outcomes of metabolic diseases.

As an antioxidant agent, Se is incorporated into selenoproteins, which play important roles in glucose and lipid metabolism. Moreover, Se shows great potential for redox regulation to maintain cellular homeostasis and metabolism [14]. Previous studies have reported that excess ROS play a role in the complex pathogenesis of metabolic diseases [13]. Therefore, this review focused on the potential role of Se in the development of metabolic diseases. As mentioned above, we systematically reviewed current data on the correlation between Se status and the risk of metabolic diseases, including CHD, HT, NAFLD, and T2DM. Surprisingly, the specific role of Se levels in metabolic diseases remains controversial. Some studies indicate that higher levels of Se have significantly beneficial effects in the prevention of CHD. By contrast, other studies have indicated a positive correlation between Se levels and T2DM. With regard to the protective action of Se in HT and NAFLD, research opinions remain inconsistent. The results of different studies highlight the complex physiological role of Se. Although the role of Se in metabolic diseases remains unclear, the antioxidant activity of Se in the pathogenesis of diseases cannot be ignored, and the molecular mechanisms underlying these paradoxical effects need to be further explored. Some studies have shown that high levels of Se reduce NO bioavailability and impair angiogenesis, and high Se concentrations induce ER stress and increase ROS accumulation, which may lead to cell apoptosis [139]. ROS can activate chemoreflex and suppress baroreflex, thereby stimulating the sympathetic nervous system and causing HT [102]. In addition, the elevated level of ROS in pancreatic *β* cells is accompanied by elevated fasting plasma insulin levels and the absence of IR, resulting in pancreatic *β* cell dysfunction and subsequent progression to T2DM [102]. These results suggest that Se may affect the redox balance in humans by regulating ROS levels, which contributes to the development of metabolic diseases. On the other hand, Cardoso et al. found that xanthine dehydrogenase (XDH) was the interacting protein that connected the pathogenesis with the molecular action of Se by searching the STITCH 4.0 and STRING databases [15]. A previous study showed an inverse correlation between GPx enzyme levels and XDH levels in diabetic rats, suggesting that Se may be related to xanthine metabolism [140]. Taken together, the mechanism underlying the role of Se in metabolic diseases, which may be dependent on or independent of the internal antioxidant defense system, should be studied in future experimental investigations.

Se is vital for many physiological processes, and adequate Se intake and status are very important for human health. Based on the importance of Se in the cellular antioxidant defense system, Se intake higher than the dietary recommendations may be protective against cancer or result in other additional health benefits which have been proposed. The therapeutic strategy of Se supplementation for metabolic diseases has been studied for many years. When studying Se supplementation in clinical trials, several aspects need to be considered, including the different types of Se used for supplementation, the level of Se at baseline in the subjects, the level of nutritional or supernutritional Se supplementation, and the duration of Se supplementation in the trial. Burk et al. noted that supplementation with SeMet and Se yeast increased plasma Se levels in a dose-dependent manner, but selenite did not [43]. Plasma Se levels were useful in monitoring the compliance and safety of Se supplementation as SeMet, but not selenite, and plasma Se levels seemed to reflect the SeMet content of yeast, but not the other yeast Se forms [43]. In addition, next-generation Se supplements, such as zerovalent Se nanoparticles (SeNPs) and selenized polysaccharides, slowly release active Se through an equilibrium reaction, which has a lower risk of Se excess supplementation due to their lower toxicity, higher bioavailability, and controlled release [141]. Since Se deficiency contributes to the risk of KD, administering Se supplements to the residents of KD-endemic areas significantly reduced the incidence of KD. Therefore, Se supplementation may be a potential strategy for KD prevention and treatment. Regarding the role of Se supplementation in metabolic diseases, although many studies have shown the protective action of Se supplementation in trials, some studies have shown that Se supplementation has no effect, even contributing to the development of CVD and T2DM. Evidence from large RCTs is needed to confirm the feasibility of Se supplementation as a potential therapy for metabolic diseases and to investigate the potential underlying mechanisms and the possibility of public health interventions.

However, supernutritional Se supplementation may result in acute or chronic Se poisoning, and the difference between potential beneficial and toxic Se level doses should be considered when recommending dosages. According to the dietary 5recommendation from the RDA, Se intake ranges from 55 to 70 *μ*g per day, which is typically based on the Se intake needed to saturate GPx activity. In general, plasma Se levels are approximately 100 *μ*g/L, and urinary Se levels range from 10 to 85 *μ*g/L in the general population [48, 49]. Mortality has been associated with blood/plasma Se levels ranging from 300 *μ*g/L to 30,000 *μ*g/L compared to normal levels of 100 *μ*g/L. As mentioned above, Se deficiency is closely related to the occurrence, development, prognosis, and outcome of many diseases, as well as the all-cause mortality rate. Therefore, the minimum requirement for Se is to prevent the prevalence of Se-deficient diseases, such as KD. In addition, owing to the toxicity of high Se levels, including acute or chronic Se poisoning, noncritical Se intake without a physician's recommendation should be urgently dissuaded. As part of a therapeutic approach, there is a need to consider its limited therapeutic range to avoid overdose and related toxicity.

To summarize, this review presents an up-to-date overview of the current understanding of Se intake and human health, including Se deficiency and Se poisoning, with an emphasis on the correlation between Se status and metabolic diseases. In addition, the prospects of Se supplementation as a therapeutic strategy for prevention of related diseases are briefly summarized and discussed. Within this context, understanding the association between Se status and human health is essential for developing effective public health policies, guiding applicable clinical practice, and counteracting health issues associated with Se deficiency. In light of the current state of this field of research, future studies on the protective action of Se in metabolic diseases and the corresponding molecular mechanisms are needed to clarify the paradoxical effects of this micronutrient.

## Figures and Tables

**Figure 1:** Outline of selenium absorption and transportation under the conditions of adequate and deficient Se supply. In general, Se is mainly obtained through the diet and absorbed via the duodenum and caecum. SEPP1, the major transport form of Se, is synthesized and secreted by the liver and transported to other tissues through systemic circulation. When Se supply is adequate, plasma SEPP1 is absorbed by apoER2 in the brain, thyroid gland, testis, and other tissues and by megalin in the kidney. When Se supply is deficient, the brain, thyroid gland, testis, and SKM retain or redistribute Se to maintain physiological function, while the levels of Se in the liver, lung, and other tissues rapidly decrease, resulting in a tissue Se hierarchy.

**Figure 2:** Graphical summary of the potential effects of the various selenoproteins in tissues and organelles. In general, Se is widely expressed in many organs, such as the thyroid gland, heart, liver, pancreas, and skeletal muscle. As an antioxidant agent, Se is incorporated into selenoproteins, which play an important role in the glucose and lipid metabolism and may be involved in metabolic disorders, including cardiovascular disease, atherosclerosis, type 2 diabetes, autoimmune thyroid disorders, and nonalcoholic fatty liver disease. In addition, selenoproteins are highly expressed in the mitochondria and endoplasmic reticulum, which indicates a close correlation between energy metabolism and selenoproteins. Furthermore, the importance of selenoproteins in antioxidant defense and anti-inflammatory capacity has been widely reported. These roles may partly contribute to the role of Se within the occurrence and development of diseases.
